# An Analysis and Research on Chinese College Students' Psychological Barriers in Oral English Output from a Cross-Cultural Perspective

This article has been retracted.

**DOI:** 10.1155/2022/2862727

**Published:** 2022-07-21

**Authors:** Shuai Zheng

**Affiliations:** College of Foreign Languages and Cultures, Chengdu University, Chengdu 610106, Sichuan, China

## Abstract

English, as China's second language, is a part of the overall quality of the people. Mastering this universal language in the world is required to communicate with the world. The most important purpose of learning a language is to communicate, and listening and speaking ability is the most important language skill. However, under the influence of the test-oriented education model, English teaching in our country places too much emphasis on the cultivation of reading and writing ability and neglects the training of oral expression ability. In this context, this research proposes an oral English teaching assistance program for both teachers and college students and plans to build an artificial-intelligence-based oral English teaching assistance system. The combination of ability and oral English teaching solves the drawbacks of traditional oral English teaching and establishes a new teaching form for college students' oral English teaching. Combined with the popular trend of Internet electronic teaching methods, it realizes a free and online platform for learners to correct and improve pronunciation, laying a certain foundation for the development of mobile online English pronunciation learning in the future and solving the psychological barriers to college students' oral English output.

## 1. Introduction

In recent years, Chinese people's enthusiasm for learning English has not declined at all, and there is a growing trend. However, among highly educated Chinese students, “dumb English” can be found everywhere, which is thought-provoking. In the stage of higher education, college students are in the superposition of multiple relationships such as personality, environment, and teachers, resulting in difficulties in oral English output. Most college students in high school are in the period of mechanical memory. There are many problems in learning English, such as rote memorization, whether they can write or read, and whether they can recognize or not. These problems in college students' oral English are not conducive to their continuous learning of English, which has attracted the attention of the majority of English educators. The mastery and application of a foreign language must meet the requirements of the four indicators of listening, speaking, reading, and writing in the language, and English is no exception. Among the four indicators, the ability to listen and speak is not only the basis for learning English well but also the guarantee for learning English well. It plays an important role in English learning. In recent years, people from all walks of life have paid more and more attention to listening and speaking ability, which has gradually aroused people's attention to oral English teaching. However, there is a fact that cannot be ignored that there are many problems in the current oral English teaching, which seriously hinder the development of students' oral English ability. In China, most teachers in all grades and stages still adopt the traditional teaching mode of “teacher speaking,” which pays too much attention to the learning of basic language knowledge, such as grammar and vocabulary, and ignores oral teaching activities. There are also many problems in the design of oral English activities, and the quality of oral English teaching needs to be improved.

The first is the lack of language environment. Although there are not many English courses in the curriculum, it cannot guarantee students' effective access to English every day. Most of the time students spend learning English is limited to a limited number of English classes. At present, schools at all levels in China mainly adopt the class teaching system, and there are a large number of students in each class, so there is no time and opportunity to ensure each student's speech, and the students outside the class lack the atmosphere of speaking English. Secondly, in terms of teaching methods, many teachers still cannot adhere to the teaching method of teaching in English. Most English teachers still use the method of explaining grammar points or other knowledge points in Chinese. In such a classroom environment, students cannot be guaranteed to have a certain amount of listening input. Without the environment, it is difficult for students to carry out effective oral English output. Moreover, students' own factors are also major factors that cause problems in oral English teaching activities. Most Chinese students are influenced by Chinese traditional thoughts and are implicit in oral communication. In addition, introverted personality and other psychological barriers make many students afraid or unwilling to speak English. This also brings some obstacles to oral teaching activities.

With the deep integration of technology and education, we are ushering in an era of intelligent education, and the traditional teaching methods are also being changed by technology. Under the current cross-cultural conditions, oral English teaching has become an indispensable part of Chinese English education. The contradiction between traditional teaching methods and oral English teaching needs is becoming increasingly prominent. The development of artificial intelligence technology will help solve this contradiction. [1–5].

## 2. Related Work

In 2001, China successfully joined the WTO. In the same year, relevant government agencies began to offer English courses in primary schools, and English has covered all stages of students' careers. The government attaches great importance to English learning. From elementary school to university, English proficiency will be assessed. English is a compulsory subject in the entrance examination. Even if you enter society, English is still the focus of many companies' recruitment. In the past, English learning focused on written test scores, which led many English learners to ignore the importance of oral pronunciation. Different from the previous English learning, in addition to focusing on the written test results, the ability of oral communication is becoming more and more important. In the 2018 National College English Test (CET-4/6), it is a good idea to officially add the oral test. However, spoken English pronunciation is largely influenced by native language (Language 1, L1) pronunciation habits. Although the official language of China is Putonghua and China is a country with abundant language and cultural resources, the existing languages (dialects) can be divided into eight major factions, with more than 100 dialects subdivided. The diversity of language and culture has led to many pronunciation problems in foreign language learning, not only in spoken English but also in Mandarin pronunciation that is also affected by dialect habits. For example, many people do not distinguish between “*n*” and “*l*” in Chinese Pinyin; the front nasal and the rear nasal are not distinguished; “zh” and “z” are not distinguished, and so on.

With the rapid development of machine learning, the field of speech recognition has also introduced this technology. From the perspective of machine learning, the pronunciation error detection of a phoneme can be regarded as a binary classification problem, that is, to determine whether the pronunciation of the phoneme is correct. Therefore, many researchers design and improve pronunciation error detection systems from the perspective of classifiers. Neri et al. compared the performance of the GOP algorithm, decision tree, and linear discriminant analysis in distinguishing consonant phonemes in Dutch [9]. The experimental results show that the recognition accuracy of linear discriminant analysis is higher than that of the GOP algorithm and decision tree. As the feature complexity becomes higher, many researchers begin to introduce support vector machine (SVM) into pronunciation error detection algorithms. By analyzing the pronunciation mode and pronunciation position of each phoneme, Li et al. classified the speech segment of each phoneme according to its GOP value and trained them separately and then trained an SVM classifier for each phoneme to detect pronunciation errors. To improve the system's ability to discriminate pronunciation quality, in recent years, deep learning has developed rapidly in the field of speech recognition, and the introduction of deep learning technology has further improved the accuracy of word recognition. In 2010, Qian et al. studied the acoustic modeling of the hybrid DBN-HMM framework in English pronunciation error detection and diagnosis. This is the first time to compare the performance of DBN-HMM with the best-tuned GMM-HMM trained on ML and MWE on the same set of features. Experiments show that the method captures speech errors better than knowledge-based and data-driven speech rules but at a higher computational cost. Li et al. studied the use of multidistribution deep neural networks (DNNs) for mispronunciation detection and diagnosis (MDD) to overcome the difficulties encountered by existing methods based on extended recognition networks (ERNs) [12]. ERNs leverage existing automatic speech recognition technology to limit the search space by including possible patterns of phonetic errors of the target word as well as canonical transcriptions. MDD is achieved by comparing the identified transcripts to the canonical transcripts, which provides a significant improvement in performance. Lee et al. used DBN instead of the Gaussian mixture model (GMM) to detect word-level mispronunciation, aligning a non-native sample with at least one native sample and extracting features describing the degree of misalignment from alignment paths and distance matrices. Replacing the system input of a fully unsupervised MFCC or Gaussian posterior with a DBN posterior shows a significant improvement in system performance [6–10]. Therefore, in the pronunciation error detection and correction system, feedback and correction opinions should be provided at least at the phoneme level so that learners can focus on the most core position, so as to effectively improve the learners' pronunciation level and solve psychological obstacles.

## 3. Related Theories and Methods

### 3.1. Automatic Pronunciation Error Detection

According to the types of pronunciation errors, phonemic pronunciation errors can be divided into prosodic errors and phonemic errors. Most of the errors in pronunciation error detection, such as phoneme misreading, missing reading, and insertion, are all phonemic errors. And the pronunciation error detection of this paper is to provide the learners with direct correction feedback, so this paper focuses more on the research on pronunciation errors caused by the non-standard pronunciation-related organs and pronunciation movements and on solving the psychological barriers to the output of spoken English [11–13].

### 3.2. Corpus

The design, recording, and transcription of the data assets included in TIMIT are done in various places. Speech recognition research including Alibaba's Dharma Academy Speech Lab is also based on LibriSpeech, and the corpus used mainly includes CSTR vctk corpus and Edinburgh University corpus. The CSTR VCTK corpus contains speech data for 109 native English speakers with different accents. Each speaker read about 400 sentences, most of which were picked from the *Herald* and *The Times*. Each speaker reads a different newspaper sentence, and each set of sentences is picked using a greedy algorithm designed to maximize contextual connections and speech coverage. The corpus data can be found in the speech accent archive. The CSTR VCTK Corpus uses the same recording equipment to record all speech data: an omnidirectional headset microphone (DPA 4035), recorded in a semianechoic chamber at the University of Edinburgh with a sampling frequency of 96 kHz. Since the corpus contains non-standard pronunciations of non-native English speakers with different accents, pronunciation issues were manually annotated by experts from the Centre for Speech Technology Research (CSTR), a collaboration with the University of Edinburgh. It is suitable for the study of pronunciation error detection in this paper, so this paper selects CSTR VCTK Corpus as the experimental corpus and collects pronunciation data on this corpus. For Chinese, there are also relatively excellent corpora in China, such as THCHS30. As a supplement to the 863 corpora, the coverage ratios of diphones and triphones are shown in Table 1. Now THCHS30 has been widely used in Chinese language recognition, pronunciation error detection, and other research [14].

### 3.3. Acoustic Features

The speech signal is a time-varying stationary signal in a short period of time, and the information it contains can be roughly divided into two categories: one is semantic information, and the other is acoustic information. Large, this paper mainly involves acoustic information, and the key information contained in acoustic features is the basis of this research. Acoustic features have a certain uniqueness, and the characteristics of the signal can be more accurately expressed by analyzing and extracting these feature parameters. Therefore, the extraction of acoustic feature parameters of speech plays an important role in the pronunciation error detection system. Usually, the acoustic features of speech can be divided into two categories: the first category is amplitude, energy, and zero-crossing rate, which are the characteristics of speech signals in the time domain. The second category is the converted frequency features, such as linear prediction coefficients (LPC), Mel-frequency cepstral coefficients (MFCC), and so on. Generally speaking, it is not easy to analyze the characteristics carried by the speech signal in the time domain, so it is usually observed by converting it from the time domain to the characteristic distribution in the frequency domain. Linear prediction coefficients, formant features, and Mel cepstral coefficients are mainly used in pronunciation error detection research. Since the transition between sampling points is relatively smooth, linear predictive analysis can use this feature of speech to predict the current or future sample value based on the *p* sampling point values in the past. Assuming that at time *n*, the sample value of the speech signal is *s*(*n*), and $\hat{s}\left(n\right)$ is the predicted value of *s*(*n*), we have

(1) $$\begin{array}{c} \hat{s}\left(n\right)=\sum_{i=1}^{p}a_{i}s\left(n-i\right). \end{array}$$

Among them, *a*_1_, *a*_2_,…*a*_p_ are linear prediction coefficients, and formula (1) is called a linear predictor. If *P* is the order of the linear predictor, its system function is as follows:

(2) $$\begin{array}{c} p\left(Z\right)=\sum_{i=1}^{p}a_{i}Z^{-i}. \end{array}$$

### 3.4. Current Sample Value *s*(*n*) and Its Linear Prediction Value $\hat{s}\left(n\right)$

*ε* is the linear prediction error. Then, *ε*(*n*) is expressed as follows:

(3) $$\begin{array}{c} \varepsilon \left(n\right)=s\left(n\right)-\hat{s}\left(n\right)=s\left(n\right)-\sum_{i=1}^{p}a_{i}s\left(n-i\right). \end{array}$$

Figure 1, taking a simple speech model as an example, *H*(*z*) is called the linear prediction error filter. The linear prediction error *ε*(*n*) can be obtained by the following transfer function *H*(*z*):

(4) $$\begin{array}{c} H\left(Z\right)=1-\sum_{i=1}^{p}a_{i}Z^{-i}. \end{array}$$

Therefore, in order to minimize the linear prediction error (*n*) under a certain criterion, *ε*, the solution to the linear prediction error filter is used to solve the linear prediction coefficients *a*_1_, *a*_2_,…*a*_p_, and this process is LPC analysis.

### 3.5. Mel-Frequency Cepstral Coefficients (MFCC)

MFCC (Mel-frequency cepstral coefficient) was proposed by Davis and Mermelstein in 1980. MFCC mimics the human speech production and auditory system. According to the theoretical research on human earphones, the hearing sensitivity of the human ear to sound waves varies with frequency. MFCC takes advantage of this feature. Since this feature is developed on the human auditory model, MFCC utilizes the human auditory model to convert the linear spectrum to a Mel-scale spectrum based on the non-linear characteristics of the frequency of the human ear. The relationship between ordinary frequency and Mel-scale frequency is

(5) $$\begin{array}{c} \text{Mel}\left(f\right)=2595\times \mathrm{lg}\left(q+\frac{f}{700}\right), \end{array}$$

where *f* is the frequency in Hz. The formula shows the relationship between linear frequency and Mel-scale frequency. It can be seen from the formula that the distribution in the low-frequency part is denser than that in the high-frequency part, which is exactly in line with the change of human hearing sensitivity with frequency feature, which is then mapped onto the cepstrum [15]. The general process of MFCC extraction is shown in Figure 2.

### 3.6. Random Forest Algorithm

#### 3.6.1. Decision Tree

In the classic process of building decision tree forests, information measures based on classical probability theory are used [16–19].

#### 3.6.2. Random Forest Principle

If a new instance is to be classified, the features of that instance are input to each decision tree in the forest. The attribute metrics used by these three decision tree algorithms are shown in Table 2 [20].

Each decision tree has the following characteristics:

1. If *N* is the number of instances in the data set, then RF selects a random sample from the original data, replacing *N* instances. This instance will serve as a training set for building a decision tree forest.
2. If *M* is the number of features in the dataset, then specifying *m* features determines the splitting criterion *m* < *M*. During random forest construction, the value of *m* remains unchanged.
3. At each node of the tree: randomly select *m* features from *M* original features. Then the split criterion is calculated based on these *m* features. Subnodes are generated from top to bottom, and the splitting stops when the metric features are not improved or the data set is no longer separable.
4. No pruning is required after building each decision tree. In the beginning, Quinlan proposed the ID3 decision tree algorithm. Later, through continuous improvement, he and other researchers successively proposed the C4.5 algorithm and the CATR algorithm.

Although different attribute measures are selected, the same is that ID3, C4.5, and CATR algorithms use top-down greedy algorithms to construct decision trees, but there is no absolute good or bad for these decision tree algorithms. It is necessary to choose the appropriate decision tree algorithm according to the example and experience.

## 4. Construction of the Pronunciation Error Detection Model Based on MFCC-RF and Analysis of Experimental Results

Automatic pronunciation error detection is a means of marking the acoustic feature information hidden in the audio of standard pronunciation and non-standard pronunciation. Pronunciation error detection, especially with the rapid development of speech recognition technology in recent years, has received more and more attention from researchers. Pronunciation error detection and feedback correction in computer-aided oral language training complement each other. Pronunciation error detection is not only for detecting errors but also for providing learners with good corrective opinions and improving their pronunciation ability. The problem is that first of all, the coverage of the types of pronunciation errors is small, and the types of error detection are very limited. Then, the importance of corrective feedback is ignored. At this stage, most researches are only focused on how to detect pronunciation errors. It can indicate that the learner has problems with pronunciation and cannot put forward targeted improvement suggestions for pronunciation errors. It has little effect on the learners' ability to improve pronunciation. In order to solve the above problems, this chapter proposes a new pronunciation error detection model, which uses the Mel-frequency cepstral coefficient (MFCC) and random forest (RF) algorithm to detect the location of the pronunciation-related organs (tongue) and pronunciation errors caused by non-standard movements, and pronunciation durations are classified and detected to clarify the learners' pronunciation problems, making it a reality to provide feedback and corrections for different types of errors.

### 4.1. Problem Description and Model Evaluation

#### 4.1.1. Problem Description

In second language learning, learners are often affected by the habitual pronunciation movements of the native language, resulting in non-standard tongue positions and improper control of the pronunciation time of some phonemes. These reasons can lead to many pronunciation problems for learners.  Figure 3 is the tongue map of the standard vowel pronunciation given by the International Phonetic Alphabet (IPA). Once the learner is practicing pronunciation, if the pronunciation action does not meet the standard requirements, the pronunciation will be wrong. In the primary and secondary school classrooms, some teachers also put forward requirements on the pronunciation action of the students. For example, in the pronunciation of the Chinese pinyin letter “o,” Let the students open in a circle, but the classroom teaching teachers are one-to-many, and it is difficult to ensure that each student's pronunciation can be helped and guided. Moreover, learners often can only read and follow pronunciation through blind imitation, unaware of their own pronunciation problems, and there is no way to talk about correcting pronunciation problems. Therefore, a pronunciation error detection model based on MFCC-RF is proposed to detect the pronunciation action problem during automatic pronunciation error detection. The pronunciation classification error detection model is constructed and verified by using the pronunciation error data manually marked by the phonetic experts in the corpus [21].

#### 4.1.2. Evaluation of Pronunciation Error Detection Model Based on MFCC-RF

In pronunciation error detection and many other natural language processing studies, the selection of acoustic features is very important. Acoustic features contain phonetics and acoustic information, which is the first step for any language processing project and the foundation of the entire project. Among them, speech studies based on formants, linear prediction coefficients (LPC) and Mel-frequency cepstral coefficients (MFCC) are the most extensive. In the research of this automatic pronunciation error detection system, the requirements for antinoise interference are relatively high. It is necessary to reduce the noise of the input model features as much as possible and include as much information contained in the learners' pronunciation as possible, so as to eliminate the lack of features and improve the accuracy of error detection. Among these acoustic features, the formant estimation feature contains less information, and the Mel-frequency cepstral coefficient is better than the linear prediction coefficient in signal stability, and it can also maintain a good performance when the signal-to-noise ratio is reduced. Therefore, this paper chooses the Mel-frequency cepstral coefficient as the feature input of the machine learning algorithm model.

Random forest is an extremely widely used algorithm. In the more than 20 years since it was proposed, the random forest algorithm has been used in many fields such as image recognition, stock prediction, and e-commerce and achieved good results. One of the advantages of random forest is that it can be used for classification because its basic unit is a decision tree. By building multiple decision trees and then merging these decision trees together, each decision tree gives a result. The mode of voting determines the final classification result. Due to the random sampling and replacement strategy, the training model error can be reduced and the generalization ability is better than other machine learning algorithms.

### 4.2. Framework of the Pronunciation Error Detection Model Based on MFCC-RF

Figure 4 shows the flow chart of the pronunciation error detection model algorithm based on MFCC-RF. The left part of Figure 4 is the data collection and acoustic feature extraction process. On the right is the model training optimization and test validation part. As shown in Figure 4, in the construction of the pronunciation error detection model based on MFCC-RF, the steps are as follows.

#### 4.2.1. Step 1: Preprocessing

The preprocessing part includes forced text alignment and phoneme separation of speech data:

  The data obtained from the speech corpus is the whole sentence audio data file. The Hidden Markov Model Toolkit (HTK) is used to force-align the audio file with the reference text (Force-Alignment).
  Obtain the alignment time information at the phoneme level by forcing alignment and cut and separate it according to the phoneme alignment time information to obtain phoneme data.

#### 4.2.2. Step 2

In acoustic feature extraction, the phoneme data obtained in the first step are extracted for MFCC acoustic features. In this paper, a total of 13-dimensional MFCC plus 13-dimensional first-order difference and 13-dimensional second-order difference coefficients are extracted to form a total of 39 dimensions.

#### 4.2.3. Step 3: Data Set Preprocessing

This part mainly includes dividing the acquired feature data set into a training data set and a test data set and normalizing them. The normalization is for automatic pronunciation error detection features. The data is limited to a certain range; the purpose is to reduce the difference of the data by reducing the discrete degree of the automatic pronunciation error detection feature data so that the fluctuation of the data is limited to a certain range; and the normalization operation has no effect on the original distribution of the data. This paper chooses the linear function transformation normalization method.

Random forest model used the 39-dimensional MFCC feature vector of the training data set as input. The default initial model parameters, generally the default parameters of random forest, can obtain better classification accuracy, but this paper still chooses cross-validation to tune the parameters.

#### 4.2.4. Step 4

The test set of pronunciation error detection feature data is used to test the pronunciation error detection classification model established by the algorithm. The accuracy of pronunciation misclassification detection is obtained. The optimal model is further determined by the evaluation index. The evaluation metrics in this paper are calculated based on a confusion matrix, where mispronunciation detection can produce six types of results: (1) correct accept (CA), that is, the number of correct pronunciations judged to be correct; (2) false refuse (FR), that is, the number of correct pronunciations judged as the current mispronunciation type; (3) correct other (CO), that is, the number of correct pronunciations judged to be other mispronounced types; (4) correctly rejected (correct refuse, CR), that is, the current pronunciation error type is judged as the number of the current pronunciation error class; (5) error acceptance (false accept, FA), that is, the number of the current wrong pronunciation type judged as the correct pronunciation type; and (6) false other (FO) that means the current pronunciation wrong type is judged as the number of other pronunciation wrong types.

#### 4.2.5. Step 7

This step presents the calculation of evaluation indicators. According to the confusion matrix, common indicators for evaluating the constructed model can be obtained. This paper selects the following types:

(1) Accuracy: it is the degree of accuracy of the correct pronunciation type in the sample.
  (6) $$\begin{array}{c} \text{Accuracy}=\frac{\text{CR}+\text{CA}}{\text{CR}+\text{FA}+\text{FO}+\text{CA}+\text{FR}+\text{CO}}. \end{array}$$
(2) Recall rate: the probability that the current mispronunciation type is correctly judged as the current mispronunciation type.
  (7) $$\begin{array}{c} \text{Recall}=\frac{\text{CR}}{\text{CR}+\text{FA}+\text{CO}}. \end{array}$$
(3) False alarm rate: it is the probability that the current pronunciation error type is judged as the correct pronunciation type.
  (8) $$\begin{array}{c} \text{FA rate}=\frac{\text{FA}}{\text{CR}+\text{FA}+\text{CO}}. \end{array}$$

### 4.3. Data Set Acquisition

#### 4.3.1. Forced Alignment and Phoneme Separation

The corpus used in this study is the CSTR VCTK Corpus of the University of Edinburgh. The selected data comes from the speech data manually annotated by phonetics experts from the Speech Accent Archive. The pronunciation error detection in this paper is carried out at the phoneme level, so first of all, the speech should be forced to be aligned to the phoneme level, and the time information should be found to separate the pronunciation phonemes. The forced alignment process is done with the help of the HTK toolkit. HTK is a toolbox developed by the Cambridge University Department of Engineering (CUED) for speech recognition research, the full name of which is the Hidden Markov Model Toolbox.

The forced alignment steps are described as follows:

1. The text file is processed with special punctuation marks, and the English word segmentation process is finally saved in UTF-8 format.
2. The audio file is converted into a monophonic format with a sampling rate of 16,000 Hz, and the starting and ending points of the speech are accurately detected through endpoint detection processing.
3. The reference text is mapped from words to sounds. According to the speech recognition model in the HTK toolkit, the word-sound space is aligned frame by frame through the posterior probability of the hidden Markov state sequence.
4. Dynamic warping Viterbi alignment is used for each frame of data.

Figures 5(a) and 5(b) are the spectrograms of the word please before and after the pronunciation alignment, respectively.

Speech and text-aligned temporal information of the output sentence by forced alignment. According to the output voice and text alignment time information, read the phoneme separation level of the text grid, obtain the start time and end time of a phoneme in the phoneme level, and cut the phoneme to obtain the pronunciation phoneme.

#### 4.3.2. MFCC Acoustic Feature Extraction

The FBank feature is very similar to the MFCC feature. For the audio information, the FBank feature retains more original information, and the feature dimension is larger than that of the MFCC. When the FBank is filtered by the filter bank, there is an overlapping area between adjacent filter banks. Therefore, the correlation between its features is relatively high, and deep learning speech detection requires a good degree of discrimination, so it can be concluded that the FBank algorithm is not suitable. It has been studied that MFCC has excellent classification and recognition performance in the field of audio research in deep learning, which is inseparable from the excellent discrimination of MFCC. At the same time, the non-linear relationship expressed by MFCC is similar to the human auditory system, so it can well reflect the auditory characteristics of the human ear, which is very suitable for speech detection and error correction research. To sum up, this paper selects the MFCC feature extraction algorithm among the three common audio feature extraction algorithms and expresses the audio features with MFCC. In the preprocessing stage, MFCC feature extraction has undergone operations such as preemphasis, framing, and Hamming window addition. The following will continue to perform feature extraction on the preprocessed signals. First, perform Fourier transform on the preprocessed audio signal.  Figure 6 shows the waveform of the original signal. The *x*-axis corresponds to the sampling point, and *y* represents the sound amplitude.  Figure 7 is the frequency spectrum of the speech signal after the Fourier transform.

After the preprocessed audio signal is Fourier transformed, it needs to pass through the Mel filter bank. As shown in Figure 8, it is a Mel filter bank composed of 26 triangular filters. From the graph of the Mel filter bank, it can be seen that there is an obvious overlap between adjacent triangular filters, which means that there is more correlation between the signal features.

Through the above discrete Fourier transform, the 13-dimensional MFCC coefficients can be obtained, and then the 39-dimensional MFCC eigenvectors can be obtained through first- and second-order difference calculations.

### 4.4. Model Parameter Settings

#### 4.4.1. Data Set Preprocessing

In order to verify the error detection performance of the model, this paper creates an audio-video test set based on mispronunciation, which contains 346 mispronounced words. The test set is mainly for /aa/, /ao/, /ow/, /ay/, /aw/, /oy/, /iy/, /ih/, /ey/, /eh/, and /ae/. The 14 phonemes uh/, /uw/, and /ah/are mispronounced. According to the lip characteristics, these phonemes can be divided into two categories: rounded and flattened, as shown in Table 3. One type of pronunciation error that this article focuses on is the pronunciation of rounded labial sounds; for example, /ey/ is misread as /aa/ as chase, /ah/ as /ao/ as away, /ae/ as /aa/ as gad, in addition to other pronunciation errors, such as phoneme addition, phoneme omission, and so on. The collected data set is normalized to reduce the difference in automatic pronunciation error detection feature data from the largest Chengdu. The linear function transformation normalization is shown in the following formula:

(9) $$\begin{array}{c} b=\frac{a-a_{\min}}{a_{\max}-a_{\min}}, \end{array}$$

where *a* is the eigenvalue of pronunciation error detection MFCC before normalization, *b* is the eigenvalue of pronunciation error detection MFCC after normalization, *a*_min_ is the minimum value in the group of pronunciation error detection MFCC features, and *a*_max_ is the group of pronunciation error detection MFCC features.

#### 4.4.2. Algorithm Parameter Setting

The random forest construction process is shown in Figure 9.

In this study, the dimension of the feature vector is moderate, and the decision tree does not need to limit the depth of the subtree when building the subtree, so the maximum depth of the decision tree max_depth is set to the default value.

### 4.5. Analysis and Comparison of Experimental Results

After testing the trained MFCC-RF model on the test set, the test set shows that the classification error detection accuracy of the test set is shown in Figure 10.

The accuracy of classification error detection for three types of errors (rising, lowing, and shorting) is verified through the test set. It can be seen that when the other parameters are optimal, for the lowing type error, it can be considered that when the number of subtrees in the random forest is 15, the classification error detection accuracy is the highest. For rising type error, when the number of subtrees in the random forest is 18, the classification error detection accuracy is the highest. Shorting type errors have the highest classification error detection accuracy when the subtree is 11. It can also be seen from Figure 10 that the error detection rate of a single decision tree for pronunciation classification error detection is about 50%, indicating that the use of a single decision tree for pronunciation classification error detection is generally effective. When the number of decision trees in the forest increases When the error detection rate of pronunciation classification continues to rise, the results given by each decision tree in the multiple decision tree forest classification model are used to vote, and finally, the classification results are determined by the mode of the subtree votes through the idea of ensemble learning to improve pronunciation classification. Therefore, in terms of the overall effect of phoneme pronunciation error detection, the MFCC-RF-based model can achieve about 80% error detection accuracy in three types of misclassifications. The classification error detection effect is better. In the test set validation, the classification error detection accuracy of ID3, C4.5, and CART decision tree algorithms and the algorithm performance (training time) during cross-validation were compared. Results are provided in Table 3.

From the results in Table 3, we can see that for the two types of errors of raised tongue position and low tongue position, the C4.5 decision tree algorithm has the highest classification error detection accuracy, but it takes the most time in cross-validation, achieving 17.6 seconds and 15.5 seconds. As for the pronunciation errors of the phoneme elongated category, when using the CART algorithm and the ID3 algorithm, the classification error detection accuracy is not much different. Among the three decision tree algorithms, the optimal training time is the CART algorithm. For the test set error, the best performing algorithm is the ID3 decision tree algorithm. There is no significant difference in the classification error detection rate of the three pronunciation errors, which is stable between 75% and 85% in each test.

## 5. Conclusion

Current research has found that college students do have barriers to oral English output, and this barrier is manifested in both verbal and non-verbal aspects. The core of computer-aided pronunciation training is pronunciation error detection and feedback correction. Because the previous pronunciation error detection focused on typical errors such as phoneme insertion, misreading, and missing reading, there were very few errors in the learners' pronunciation actions. In order to improve the learners' pronunciation more intuitively, the pronunciation error detection model constructed in this paper combined with the machine learning algorithm fills the gap in pronunciation action error detection. By selecting the acoustic features and corpus suitable for this paper, an error detection model method for pronunciation classification based on MFCC-RF is proposed. Using the acoustic information carried by the acoustic features as the distinguishing feature, the random forest classifier is trained to classify and detect the most common mispronunciation types. The experimental results show that the model can accurately identify the mispronounced phonemes. It provides a new method for automatic pronunciation error detection. Solve the psychological barriers to college students' oral English output.

## Figures and Tables

**Figure 1:** Error filter.

**Figure 2:** Mel cepstral coefficient extraction flow chart.

**Figure 3:** IPA standard vowel pronunciation tongue map.

**Figure 4:** Flow chart of the pronunciation error detection model based on MFCC-RF.

**Figure 5:** Pronunciation spectrogram of the word please: (a) before and (b) after alignment.

**Figure 6:** Original signal waveform.

**Figure 7:** Spectrogram after fast Fourier transform.

**Figure 8:** Mel filter bank.

**Figure 9:** Flow chart of the random forest construction model.

**Figure 10:** Classification and error detection results of the test set.

**Table 1:** Comparison of phoneme coverage between THCS30 and 863 corpora.

Corpus	863 corpus	THCHS30	863 + THCHS30
Number of sentences	1,500	1,000	2,500
Diphone coverage	58.4%	71.5%	73.4%
Triphone coverage	7.1%	14.3%	16.8%

**Table 2:** Metrics of three decision tree algorithms.

Algorithm	ID3	C4.5	CATR
Metrics	Information increment	Information gain ratio	Nikki index

**Table 3:** Accuracy and performance comparison of three algorithms.

Algorithm	Category			
	Performance	Rising	Lowing	Shorting
ID3	Accuracy (%)	7 5.5	7 8.5	8 2
	Training time (s)	1 5.46	1 5.0	1 7.32
	Test set error (%)	5.7 _	4.4 _	3.6 _

C4.5	Accuracy (%)	8 6.6	8 1.5	7 7.5
	Training time (s)	1 7.6	1 5.5	1 3.8
	Test set error (%)	7.2 _	7.86 _	5.6 _

CART	Accuracy (%)	8 5	7 9.5	8 2.5
	Training time (s)	1 2.37	1 4.25	1 1.68
	Test set error (%)	8.0 _	7.62 _	7.05 _

## Data Availability

The data set can be accessed upon request to the author.
